# Effect of Risk-Focused Diversified Safety Management Mode in Patients with Major Artery Stent Implantation

This article has been retracted.

**DOI:** 10.1155/2022/1284254

**Published:** 2022-09-30

**Authors:** Yan Shao, Cai-Juan Wu, Youjun Mao, Dong-Mei Li, Yun-Zhou Wang, Kang Zhu

**Affiliations:** Changzhou 2nd Hospital, Vascular Surgery, Changzhou 213164, China

## Abstract

**Background:**

Intracranial atherosclerotic stenosis (ICAS) causes a series of neurological symptoms, such as vertigo, impaired consciousness, limb weakness, ataxia, dysphagia, ocular motility disorders, and visual impairment. With the improvement of people's living standards, there are higher requirements for nursing care. Nursing, as an indispensable part of medical care, is closely related to achieving the goal of patient's safety and the overall quality of nurses, quality of care, and nursing management methods.

**Objective:**

To explore the effect of risk-centered diversified safety management in patients undergoing aortic stenting.

**Methods:**

Eighty patients with cerebral infarction were selected and treated with percutaneous transluminal angioplasty and stent implantation (PTAS). Then they were divided into a control group (40 cases) with routine monitoring and an experimental group (40 cases) with risk-focused intervention of a diversified safety management model according to the mode of care. Patient satisfaction and blood index test results were compared after the intervention.

**Results:**

Patients in the experimental group had 6 falls, 3 bed falls, 3 phlebitis, 4 tube slips, and 10 deep vein thrombosis, all significantly fewer than those in the control group. Thirty-eight patients in the experimental group expressed satisfaction with safe management, which was substantially better than the control group (*P* < 0.05). The levels of tissue plasminogen activator (tPA), plasminogen activator inhibitor-1 (PA1-1), and von Willebrand factor (vWF) in the experimental group were (13.5 ± 1.3) ng/mL, (60.1 ± 9.9) ng/mL, and (2.1 ± 0.2), respectively, which were substantially lower than those in the control group ((14.6 ± 2.4) ng/mL, (64.2 ± 10.7) ng/mL, and (2.8 ± 0.3)), respectively (*P* < 0.05).

**Conclusion:**

The risk-centered diversified safety management model can effectively reduce the probability of adverse events in patients, improve patient satisfaction with nursing services, and promote faster postoperative recovery, which has clinical application value.

## 1. Introduction

The primary cause of ischemic cerebrovascular disease and transient ischemic attack (TIA) in China is intracranial atherosclerotic stenosis (ICAS) [1, 2]. The results of the 2014 CICAS study showed that 46.6% of patients with ischemic stroke and TIA in China had atherosclerosis and that patients with combined ICAS had severe symptoms and a high recurrence rate during the follow-up period [3, 4]. Therefore, effective treatment of ICAS has received a lot of attention from neurologists in China.

Currently, the main treatments for ICAS include pharmacological therapy, endovascular therapy, and intracranial and extracranial arterial bypass grafting. In recent years, endovascular treatment has gained attention because of its minimally invasive and rapid recovery characteristics, but the results of the SAMMPRIS study and the VISSIT study suggest that the incidence of the primary endpoint event (stroke and death within 30 d of enrollment) in the endovascular treatment group was 14.7%, which far exceeded the incidence of 5.8% in the drug group [5, 6]. As the SAMMPRIS study has been questioned in various aspects regarding operator experience and enrolled cases, it has been explored accordingly in China. The results of a multicenter registry study of stenting for symptomatic intracranial artery stenosis in China, led by Tiantan Hospital, showed that the perioperative endpoint event rate for endovascular treatment of patients with symptomatic ICAS after rigorous screening was 4.3% [7, 8], which was much lower than the complication rate in the stent group of the SAMMPRIS study. The results of the CASSISS study, led by Xuanwu Hospital, will be available in 2015, which also excluded complex lesions >14 mm in length [9, 10]. With the continuous improvement of modern medical imaging techniques and adjuvant treatment materials, percutaneous transluminal angioplasty and stenting (PTAS) has gradually become available to the general public. It has now been developed as a new method for the treatment of sclerotic stenosis of large intracranial arteries. Relevant clinical studies have shown that patients with asymptomatic intracranial large artery stenosis treated with PTAS of the intracranial arteries have a significantly lower probability of postoperative stroke and better long-term outcomes, which is conducive to improving the prognosis of patients [11, 12].

Nursing, as an indispensable part of medical care, is closely related to the overall quality of nurses, nursing quality, and nursing management methods and is related to the achievement of patient safety goals [13, 14]. In recent years, the safety of patients during hospital treatment has become an important issue of general concern at home and abroad. Foreign research on this issue started earlier and is more in-depth, with many relevant studies and relatively perfect research results. The important research directions of nursing risk management abroad mainly include the incidence of nursing risk accidents, the concept of patient safety, and relevant safety measures. According to the prevalence and seriousness of patient safety problems, foreign scholars actively analyze and explore their causes and propose targeted measures. At this stage, some developed countries have begun to pay attention to the training of medical staff in patient safety education knowledge and have constructed a content system for patient safety education [15, 16]. Diversity management is a human resource management activity, the basic principle of which is to recognize different problems in the work and adopt different methods to help solve them [17, 18]. It can reach all aspects of the work and continuously improve the hidden problems in each of them, helping to improve the effectiveness of care.

Therefore, 80 patients with cerebral infarction were selected for PTAS of the intracranial artery, and routine care and diverse risk-focused safety management were given during the procedure. The intervention lasted for one month, and the changes in the indicators after the intervention were recorded. The effects of the risk-focused diversified safety management in patients undergoing PTAS surgery of large arteries were compared and analyzed, hoping to provide reference values for its future clinical application.

## 2. Materials and Methods

### 2.1. The Research Object

A total of 80 patients with cerebral infarction aged 18-75 years who received treatment in our hospital from January 2020 to May 2022 were selected. The two groups were divided according to whether the diversified risk-focused safety management mode intervention was carried out after PTAS. The control group (40 cases) received routine monitoring, and the experimental group (40 cases) received the risk-focused diversified safety management mode intervention. Inclusion criteria are as follows: I. Patients with cerebral infarction confirmed by CT or MRI diagnosis on admission; II. No serious heart, liver, or renal insufficiency; III. No rheumatic heart disease, atrial fibrillation, blood system, or autoimmune diseases; IV. No drugs affecting coagulation function within one month; V. No history of major brain injury or surgery and no history of active hemorrhagic disease; VI. Cerebrovascular DSA confirmed intracranial arterial stenosis ≥50%. Exclusion criteria are as follows: I. Patients with transient cerebral ischemia; II. Chronic complete occlusion or severe calcification of intracranial arteries; III. Stenosis or occlusion of the middle cerebral artery, distal anterior cerebral artery, and posterior cerebral artery; IV. Neurological dysfunction after severe stroke (NIHSS score [19, 20] more than 4 or consciousness disorder); V. People allergic to contrast agent.

The experimental procedure was approved by our ethics committee, and written informed consent was obtained from all subjects included in the study.

### 2.2. Treatment Measures

DSA examination was as follows: most subjects underwent routine preoperative examination after admission. Food was forbidden four hours before surgery, and the patient was sent to the Cath lab for total cerebral angiography under local anesthesia. After a successful femoral artery puncture by the Seldinger method, a 6F arterial sheath was inserted, and angiography was performed on the aortic arch, internal carotid artery, bilateral common carotid artery, subclavian artery, and vertebral artery. At the same time, the front and side positions were continuously exposed until the veins were empty. For suspicious vascular lesions that could not be identified by conventional projection, multiangle angiography was continued. The WASID equation [21] was used to calculate the degree of intracranial arterial stenosis: stenosis rate % = [1 − (*D*_stenosis_/*D*_constant_)] × 100%. *D*_stenosis_ refers to the diameter of the smallest vessel in the stenosis segment, and *D*_constant_ refers to the diameter of the proximal artery in the stenosis segment. The measured rates of arterial stenosis were determined by two experienced neurointerventionists who read the films independently.

All patients underwent percutaneous endovascular stent implantation (PTAS). Postoperative blood pressure management was that the systolic blood pressure was maintained for severe stenosis between 100 and 130 mmHg, and systolic pressure was maintained in patients with nonsevere stenosis between 110 and 140 mmHg. Clopidogrel 75 mg/d and aspirin 100 mg/d were given orally for 12-16 weeks, followed by aspirin 100 mg/d for continuous treatment.

### 2.3. Risk Management Methods

- Recognition period. The cases of falling/falling in bed, deep vein thrombosis, accidental burns, medication errors, phlebitis, and qualified rate of transport and handover were recorded. All risk factors related to objective patient safety management during treatment were sorted, and inspection tables were constructed. The number of cases of projects related to objective patient safety management that occurred in each clinical department was noted in detail. Indicators related to the management of patient safety objectives were screened. The nursing risk management projects in technology, service, business, and management were comprehensively counted from the perspectives of human, machine, material, environment, and law.
- Evaluation Period. Questionnaires were issued, and statistical analysis was conducted on all risk management projects. The risk index (number of occurrences × severity × discovery) was determined. A score of more than 350 was classified as unacceptable risk, 100-349 as major risk, 35-99 as moderate risk, 10-34 as permissible risk, and 1-9 as negligible risk. According to the statistical results, the checklist and Plato were formulated, and the patient safety objective risk management items were determined according to rules 20 and 80.
- Coping period. From the management aspect, the first is to run the nursing risk assessment scale comprehensively. Four nursing risk assessment scales were constructed and improved, including the risk factor assessment record for preventing patients from falling/falling in bed, the risk factor assessment scale for preventing catheter slip, the risk factor assessment scale for preventing phlebitis, and the risk factor assessment scale for preventing deep vein thrombosis. Through trial, revision, training, pilot, comprehensive rollout, and other management means, a comprehensive assessment of patients was implemented, which aimed to reduce or eliminate the incidence of falling/falling in bed, catheter shedding, phlebitis, and other items that affect the patient safety objectives and effectively ensure patient safety. Second, all relevant systems, processes, standards, and plans were enhanced for the implementation of patient safety objectives, such as the establishment of management systems, processes, standards, and plans for preventing patients from falling/falling in bed, preventing patients from phlebitis, and preventing pipeline slippage and deep vein thrombosis standard operation instructions (SOPs). A patient safety management system and assessment standards were established, as did the core monitoring index and key department management monitoring index of the whole hospital inpatient safety management. The nursing work notification system and health education system of various patient safety objectives were optimized and implemented. The third is to strengthen and implement oversight. The system and standard for verification, supervision, guidance, and evaluation of special risk projects of nursing management departments at all levels were established. Continuous improvement of care quality was carried out through PDCA quality management tools. A hospital-level comprehensive CQI nursing quality management project was established to strengthen the implementation and implementation of patient safety objectives and ensure effective management. From the aspect of personnel management, the implementation of training work was strengthened, and training plans were improved. Systematic and comprehensive training and assessment of the newly built specifications were conducted to ensure unified mastery and consistent execution of the working standards. In terms of facilities and environment, various warning labels should be established and improved to ensure patient safety, such as antifall/falling in bed, careful sliding, careful stepping, careful breaking of road, careful use of sugar, turning over card, antiscald, anticatheter falling off, careful electric shock, high-risk drugs, easily confused drugs, and other safety management labels. In terms of articles, all kinds of safe and qualified articles were provided, including all kinds of disposable articles, sterile articles, and implanted articles. In terms of equipment, operation procedures, troubleshooting, and emergency plans were established for various instruments and equipment, and training was implemented in a planned way to ensure that the efficiency of all staff was 100%.
- Monitoring period. Risk project quality inspection standards and evaluation standards were developed, and comprehensive organizational inspection, supervision, and evaluation of nursing work were planned to carry out the risk management and implementation effect. A comprehensive summary of project risk management achievements was made. The existing deficiencies should be carefully analyzed, improved, and implemented to make continuous quality progress and ensure the unification of standards. The implementation of specific norms as well as the realization of key projects, important standards, key norms, homogeneous management, and implementation were also important.
- Filing Period. Through comprehensive implementation, patients' safety objectives were fully collected and sorted out, and successful measures and methods were consolidated. A series of nursing risk management project case collections and standard operation protocols (SOPs) were set up to solidify and implement the project. All nursing colleagues in the hospital were educated and warned to prevent risks and learn and improve together.

### 2.4. Observation Indicators

- Management effectiveness evaluation. A questionnaire survey was used to evaluate the satisfaction with safety management and other contents of inpatients one month after the intervention. The Inpatient Safety Management Satisfaction Scale was mainly developed according to the Inpatient Satisfaction Scale, relevant literature, and specific work practice and has good reliability and validity.
- Blood index test. Two-milliliter venous blood samples were collected on an empty stomach at 7:00 am before the intervention and after the intervention experiment. Plasma was separated by centrifugation within 1 h (3000 RPM, 10 min, 20°C), and the upper plasma was divided into a 0.5 mL EP tube, which was numbered according to the collection date and stored in a low-temperature refrigerator at −70°C for examination.

The detection principle was as follows: quantitative determination of target antigen levels was conducted by the ELISA double antibody sandwich method. The coated antitarget antigen-antibody was combined with the target antigen in the plasma to be tested, and the enzyme-conjugated antibody was added to form a complex, which reacted with the substrate to display color. The A value measured at 490 nm was proportional to the plasma antigen content to be measured. According to the corresponding standard point data, the standard curve was drawn in Excel, and the standard curve equation was established. The concentrations of tissue plasminogen activator (tPA), plasminogen activator inhibitor-1 (PA1-1), and von Willebrand factor (vWF) in the samples to be tested were calculated by the standard curve equation. Normal plasma concentrations of tPA and PAI-1 are 1.0-12.0 ng/mL and L5∼45 ng/mL, respectively. The plasma vWF level was measured as its ratio to the standard plasma content, and the normal range was 60%-150% or 0.6-1.5.

### 2.5. Postoperative Care

#### 2.5.1. Close Observation of Vital Signs

Patients were admitted to the intensive care unit directly after surgery and were given intensive care with continuous monitoring of several parameters and close observation of changes in vital signs. Blood pressure was measured every 5-10 min during the 24 hours after surgery, and once an hour after the blood pressure stabilized for 24 h. The patient's consciousness, pupils, speech and body movement, and the presence of severe headache were observed at any time, and the doctor was notified of any abnormalities to prevent complications.

#### 2.5.2. Prevention of Arterial Embolism and Bleeding in the Lower Extremity

After Wingspan stenting, the puncture site is usually sutured intravascularly with a vascular suture, but the suture may fail due to the influence of the technique, and the arterial pulsation and color of the punctured limb should be noted. Therefore, the pulsation and skin color of the dorsalis pedis artery on the operated side should be closely observed, and the dorsalis pedis artery should be measured every 30 min for 6 consecutive times. If the pulsation of the dorsalis pedis artery is significantly weaker than that of the opposite side and the pain of the lower limb is obvious after the operation, and the skin color is cyanotic, it indicates the possibility of arterial embolism of the lower limb. No lower limb artery embolism occurred in this group, but there were two cases of bleeding at the puncture site.

#### 2.5.3. Application of Postoperative Anticoagulant Drugs

The application of postoperative anticoagulant drugs is directly related to the success or failure of surgery. The most dangerous postoperative complication is acute arterial occlusion, which is mainly caused by subplaque bleeding or secondary thrombosis after plaque rupture. Therefore, postoperative treatment with low-molecular weight heparin is routinely administered, and patients are given warfarin 0.4 mLq 12 h subcutaneously for 1 week, aspirin 100 mg, and plavix 75 mg orally according to the doctor's prescription after returning to the ward. During the period of anticoagulation, the clotting situation was closely observed, and the clotting time and prothrombin time were monitored after the operation. The skin mucosa was closely observed for bleeding spots or purpura, the color of urine and stool, and other organs for signs of bleeding.

### 2.6. Statistical Methods

Data were processed and analyzed by SPSS 22.0. The counting data were expressed as the rate (%), while measurement data were expressed as the mean ± standard deviation ($\bar{x}\pm s$). The differences between the two groups were compared by *T* test, and continuous indicator groups were compared by analysis of variance. *P* < 0.05 was considered statistically significant.

## 3. Results

### 3.1. Basic Information of the Research Subjects

Eighty patients with cerebral infarction were randomly divided into the experimental group and the control group, with 40 in each group. In the experimental group, there were 16 males and 24 females, with an average age of 55.3 ± 2.7 years. After preoperative examination, there were 18 cases of severe stenosis and 21 cases of nonsevere stenosis, while in the control group, there were 15 males and 25 females, with an average age of 56.4 ± 3.1 years. There were 22 cases of severe stenosis and 19 cases of nonsevere stenosis. There was no considerable difference in basic data between the two groups (*P* > 0.05) (Table 1).

### 3.2. The Incidence of Adverse Events in the Two Groups

Statistically, there was no remarkable difference in unsafe events in postoperative transport between the two groups (*P* > 0.05). In the experimental group, there were 6 falls, 3 bed falls, 3 phlebitis, 4 pipeline slippage, and 10 deep vein thrombosis. In the control group, there were 28 falls, 22 bed falls, 14 phlebitis, 10 pipeline slippage, and 24 deep venous thrombosis. The experimental group had remarkably fewer unsafe events than the control group, and the difference between the two groups was considerable (*P* < 0.05) (Figure 1).

### 3.3. Survey Results of Patients' Satisfaction with Nursing Services

The results in Figure 2 showed that there was no statistically significant difference between the groups in the satisfaction of nursing staff with the service attitude, dress code, and operation technique (*P* > 0.05). In the experimental group, 36 patients were satisfied with the hand hygiene of nursing staff and 35 patients were satisfied with the operation standard, while in the control group, 29 patients were satisfied with the hand hygiene of nursing staff and 27 patients were satisfied with the operation standard (*P* < 0.05).

### 3.4. Investigation Results of Patients' Satisfaction with Safety Management

According to the investigation shown in Figure 3, there was no statistical significance between the two groups in terms of checking patients' information and respecting patients' privacy during nurses' operations (*P* > 0.05). Thirty-eight, 35, and 37 patients in the experimental group were satisfied with safety education, medication safety, and safety reminders, respectively, while 30, 24, and 28 patients in the control group were satisfied with safety education, medication safety, and safety reminders, respectively, with considerable differences (*P* < 0.05).

### 3.5. Overall Evaluation of Patient Satisfaction

According to the survey results, there was no great difference between the two groups in satisfaction with the nursing service arrangement (*P* > 0.05). There were 38 patients in the experimental group who were satisfied with safety management, while there were only 27 patients in the control group who were satisfied with safety management, and the difference between the two groups was considerable (*P* < 0.05) (Figure 4).

### 3.6. Results of Blood-Related Indicators of Patients

Blood test results showed no notable differences in blood tPA, PA1-1, or vWF between the two groups before postoperative intervention (Figures 5–7). After intervention, the levels of tPA, PA1-1, and vWF in the experimental group were 13.5 ± 1.3 ng/mL, 60.1 ± 9.9 ng/mL, and 2.1 ± 0.2 ng/mL, respectively. When compared with those of the control group ((14.6 ± 2.4) ng/mL, (64.2 ± 10.7) ng/mL, and (2.8 ± 0.3)), the difference was considerable (*P* < 0.05).

## 4. Discussion

Intracranial atherosclerotic stenosis (ICAS) is one of the major causes of ischemic stroke [22, 23], accounting for more than 10% of all ischemic strokes. In Asian countries, the proportion can be as high as 30% to 67%; in China, ICAS is the most common cause of ischemic stroke, and it causes more severe stroke, longer hospitalization, and a higher recurrence rate than that of other causes [24, 25]. Patients with symptomatic intracranial atherosclerotic stenosis (symptomatic ICAS, sICAS) refer to patients with ICAS who have symptoms of cerebral ischemia and have stroke recurrence and mortality rates of 12.2%-23% within 1 year [26, 27]. Randomized clinical trial Stenting versus Aggressive Medical Therapy for Intracranial Arterial Stenosis (SAMMPRIS) and CarotidOcclusion SurgeryStudy (COSS) showed that stents were given to patients with acute ischemic stroke (AIS) caused by sICAS. stroke (AIS) is not superior to intensive medical management (IMM) alone [28, 29]. By IMM, we mean controlling patients' lipids, blood pressure, and blood glucose; regulating patients' lifestyles; enforcing smoking cessation; and encouraging exercise on the top of antiplatelet therapy [30]. However, even if IMM is strictly implemented in patients with sICAS, their 1-year stroke recurrence and mortality rates are maintained at more than 10% [31].

PTAS of intracranial arteries can directly dilate the narrowed intracranial stenotic arteries and rapidly improve the blood supply to the brain tissue in the ischemic area, which has advantages that cannot be replaced by previous pharmacological antithrombotic therapy. In addition, many relevant clinical application studies have shown that it has good therapeutic effects and safety [32]. With the introduction of relevant laws and regulations and the improvement of patients' awareness of their rights, ensuring patient safety and improving patient satisfaction are the gold standards for measuring hospital quality at this stage [33]. At present, it is important to establish a perfect risk management system, comprehensively improve the awareness and ability of risk management, and enhance the safety management of risk events. In this study, risk management items were identified and a relatively standardized and reasonable risk management pathway was explored and established.

Preoperatively, we understood the detailed condition of the patient and took the initiative to introduce the advantages and purposes of this treatment to the patient and family members to reduce the pressure on the patient. After the operation, we closely observed the vital signs, paid attention to the arterial pulsation and skin color of the punctured limb, and prevented the occurrence of arterial embolism and bleeding in the lower limb. All are for routine anticoagulation drug therapy, including close monitoring of blood clotting, observation of blood pressure changes, adjustment of the speed of antihypertensive drugs at any time, observation of the patient's consciousness, pupils' speech, and limb movement; it is the use of prophylactic drugs to prevent the occurrence of cerebral vasospasm. In conclusion, early detection of changes in condition and notification to physicians for timely treatment are the keys to reducing complications and improving the success rate of surgery. In medical activities, nurses have the most opportunities to communicate and contact with patients, and the triviality and complexity of nursing operations increase the incidence of nursing risk events. After one month of safety management intervention, the probability of adverse events in the experimental group was much lower than that in the control group, and the difference between the two groups was considerable (*P* < 0.05), effectively reducing the risk of adverse events. In the process of contact with patients, etiquette service provided an effective way to express, and nurses' considerate and meticulous service was an effective way to improve service quality. The results showed that the experimental group was significantly better than the control group (*P* < 0.05). In addition, the overall satisfaction of patients in the experimental group with safety management was also much better than that of the control group, indicating that our risk-focused safety management measures were indeed effective.

## 5. Conclusion

The results show that the risk-focused diversified safety management mode can effectively reduce the incidence of adverse events in patients, improve patients' satisfaction with nursing services, and promote faster postoperative recovery of patients. However, due to limited conditions, the sample size included in this study was small, and there was no great difference in some indicators. In addition, due to the limited research time, long-term safety management intervention for patients cannot be achieved. Further research is needed. In conclusion, the risk-focused diversified safety management model can effectively improve the quality of nursing, promote patient rehabilitation, and has clinical application value.

## Figures and Tables

**Figure 1:** Comparison of occurrence of risk events. (*Note.*^*∗*^ represents a considerable difference vs. control group, *P* < 0.05).

**Figure 2:** Results of patients' satisfaction with nursing services. (*Note.*^*∗*^ represents a considerable difference vs. control group, *P* < 0.05).

**Figure 3:** Results of patient satisfaction with safety management. (*Note.*^*∗*^represents a considerable difference vs. control group, *P* < 0.05).

**Figure 4:** Results of overall patient satisfaction (*Note.*^*∗*^represents a considerable difference vs. control group, *P* < 0.05).

**Figure 5:** Comparison of tPA levels in patients' blood. (*Note.*^*∗*^represents a considerable difference vs. control group, *P* < 0.05).

**Figure 6:** Comparison of blood PA1-1 levels of patients. (*Note.*^*∗*^represents a considerable difference vs. control group, *P* < 0.05).

**Figure 7:** Comparison of vWF levels in patients' blood. (*Note.*^*∗*^ represents a considerable difference vs. control group, *P* < 0.05).

**Table 1:** General patient information.

Group	Cases	Male cases	Female cases	Age (years old)	Severe stenosis (case)	Nonsevere stenosis (case)
Experimental group	40	16	24	55.3 ± 2.7	18	21
Control group	40	15	25	56.4 ± 3.1	22	19

## Data Availability

The experimental data used to support the findings of this study are available from the corresponding author upon request.
